# A Six-Gene Signature Predicts Survival of Adenocarcinoma Type of Non-Small-Cell Lung Cancer Patients: A Comprehensive Study Based on Integrated Analysis and Weighted Gene Coexpression Network

**DOI:** 10.1155/2019/4250613

**Published:** 2019-12-04

**Authors:** Hui Xie, Conghua Xie

**Affiliations:** ^1^Department of Radiation and Medical Oncology, Zhongnan Hospital of Wuhan University, Wuhan, China; ^2^Hubei Key Laboratory of Tumor Biological Behaviors, Zhongnan Hospital of Wuhan University, Wuhan, China

## Abstract

*Background and Goals*. To identify a multigene signature model for prognosis of non-small-cell lung cancer (NSCLC) patients, we first found 2146 consensus differentially expressed genes (DEGs) in NSCLC overlapped in Gene Expression Omnibus (GEO) and TCGA lung adenocarcinoma (LUAD) datasets using integrated analysis. We constructed a weighted gene coexpression network (WGCN) using the consensus DEGs and identified the module significantly associated with pathological M stage and consisted of 61 genes. After univariate Cox regression analysis and subsequent stepwise model selection by the Akaike information criterion (AIC) and multivariate Cox hazard model analysis, an mRNA signature model which calculated prognostic score was generated: prognostic score = (−0.2491 × EXP_RRAGB_) + (−0.0679 × EXP_RSPH9_) + (−0.2317 × EXP_RPS6KL1_) + (−0.1035 × EXP_RXFP1_) + 0.1571 × EXP_RRM2_ + 0.1104 × EXP_RTL1_, where EXP is the fragments per kilobase million (FPKM) value of the mRNA included in the model. The prognostic model separated NSCLC patients in the TCGA-LUAD dataset into the low- and high-risk score groups with a median prognostic score of 0.972. Higher scores predicted higher risk. The area under ROC curve (AUC) was 0.994 or 0.776 in predicting the 1- to 10-year survival of NSCLC patients. The prognostic performance of this prognostic model was validated by an independent GSE11969 dataset of NSCLC adenocarcinoma with AUC values between 0.822 and 0.755 in predicting 1- to 10-year survival of NSCLC. These results suggested that the six-gene signature functioned as an independent biomarker to predict the overall survival of NSCLC adenocarcinoma.

## 1. Introduction

Lung cancer (LC) is one of the leading causes of cancer-associated deaths worldwide [1, 2]. Non-small-cell lung cancer (NSCLC) accounts for 85% of all lung cancer cases [3]. Approximately 50% NSCLC is adenocarcinoma and 40% NSCLC belong to squamous cell carcinoma. Complete surgical resection is the most effective therapy for patients in the early stage, and adjuvant chemotherapy (ACT) is the standard treatment for patients in stage II-III. However, the relapse and death rates remain high. A multiparameter molecular signature provides wider insights into the heterogeneous nature of cancer including NSCLC and may more reliably predict survival and benefit from chemotherapy of cancer patients than a single prognostic biomarker and/or staging system. It is important to establish prognostic gene signatures that reflect the nature of NSCLC from multiple tiers of mechanisms.

Prognostic signatures based on gene expression profiles for NSCLC have been generated in several studies. A 14-gene signature can predict survival in resected nonsquamous NSCLC [4], identify patients at high risk of mortality despite small, node-negative lung tumors [5], improve identification of patients at risk for recurrence in early-stage NSCLC [6], and predict benefit from adjuvant chemotherapy for very early stage NSCLC, which is superior over current National Comprehensive Cancer Network (NCCN) criteria at identifying high-risk patients [7]. A 15-gene signature can differentiate high- and low-risk subgroups with significantly different overall survival and is prognostic for both adenocarcinoma and squamous cell carcinoma cases [8]. GeneFx® Lung is a multigene RNA expression signature that classifies early-stage NSCLC patients as high-risk or low-risk for disease recurrence and predicts overall survival [9]. A 6-gene signature including ABCC4, ADRBK2, KLHL23, PDS5A, UHRF1, and ZNF551 is identified to be the independent prognostic factor for overall survival [10]. A 10-gene Yin Yang expression ratio signature (YMR) based on two groups of genes with opposing function significantly can separate high- and low-risk patients with stage IA or IB adenocarcinoma and squamous cell carcinomas of all stages. The YMR signature can also predict the benefit of adjuvant chemotherapy in high-risk patients with stage I NSCLC [11]. A 17-gene panel consisting of genes involved in epithelial-mesenchymal transition (EMT), hypoxia response, glycometabolism, and epigenetic modifications for non-small-cell lung cancer prognosis has recently been identified through integrative epigenomic-transcriptomic analyses. It can clearly stratify NSCLC patients with significant differences in overall survival [12]. These gene signatures contribute to preclinical and clinical treatment of NSCLC. However, additional gene signatures are needed for accurate prognosis of NSCLC because of its complexity.

In this study, we first identified genes significantly associated with pathological M stage based on weighted gene coexpression network analysis (WGCNA) using differentially expressed genes overlapped in both Gene Expression Omnibus (GEO) datasets and the TCGA-LAUD dataset. We then selected genes significantly correlated with the overall survival of NSCLC patients among above genes according to a univariate Cox regression analysis and identified a 6-gene signature for prognosis of NSCLC based on a multivariate Cox hazard model analysis. We characterized the prognostic performance of the 6-gene signature using TCGA-LAUD dataset and validated it in an independent GSE dataset of NSCLC adenocarcinoma. Our findings suggested that the 6-gene signature is a prognostic marker for NSCLC adenocarcinoma.

## 2. Methods

### 2.1. Datasets and Workflow of Data Analysis

A total of 14 Gene Expression Omnibus (GEO) datasets regarding NSCLC were collected, including GSE19188, GSE30219, GSE10072, GSE7670, GSE2514, GSE32863, GSE21933, GSE40275, GSE12472, GSE80796, GSE8500, GSE85841, GSE19027, and GSE11969. The TCGA-LUAD RNAseq data and clinical data (level 3) of the NSCLC and ANT (adjacent normal tissue) samples were downloaded from the TCGA data portal (up to June 29, 2018) (Table 1) [13–15]. These datasets were processed and analyzed by following the workflow in Figure 1. This workflow was set up based on the published literature [16, 17].

### 2.2. GEO Datasets Processing and Integrated Analysis

The 13 raw GEO datasets (GSE19188, GSE30219, GSE10072, GSE7670, GSE2514, GSE32863, GSE21933, GSE40275, GSE12472, GSE80796, GSE8500, GSE85841, and GSE19027) were subjected to a quantitative and objective quality control using the MetaQC software package according to standardized mean ranks and principal component analysis (PCA) biplots [18, 19]. The resultant GEO datasets were designated as the training set. The training dataset was processed individually using the LIMMA (linear models within the microarray analysis) software package with log_2_ transformation and annotated by converting different probe IDs to their respective gene symbols. Duplicate gene expression values were averaged. Datasets from studies that screened differentially expressed mRNAs between human NSCLC and ANT samples were selected and combined. The MetaOmics software package (http://www.pitt.edu/∼tsengweb/MetaOmicsHome.htm) was used to integrate and analyze the GEO datasets [18].

The DEGs between NSCLC and ANT were identified by analyzing the training set using the MetaDE software package by setting the mean and standard deviation (SD) filter thresholds at 10% to filter minor changes in gene expression levels [20]. Meta-analysis was performed using Fisher's method. The modified *t* test and the permutation method by summarizing −log (*P* value) across studies and running 300 permutations (*N*_Permutations_ = 300) were used to extrapolate the *P* values [21]. *P* values less than 0.05 were considered statistically significant for the DEGs. The heatmaps were generated to illustrate the expression patterns of DEGs [20].

### 2.3. TCGA-LUAD Dataset Processing and the Consensus DEGs

The TCGA-LUAD dataset was used as the test set to verify the results from the training set. Clinical information (American Joint Committee on Cancer pathological TNM stage, gender, age at initial pathological diagnosis and histological type, especially survival status, and time to latest follow-up) was screened to remove cases with incomplete clinical traits or gene expression information and resulted in 515 cases. The TCGA-LUAD DEGs were analyzed using an empirical Bayes approach within the LIMMA software package. The DEGs of the test set with a |log_2_ fold change (FC)| ≥ 0.5 and an adjusted *P* value less than 0.05 were selected for subsequent analysis. An overlapping gene set by selecting common official gene symbols in both the training and test sets was created as the consensus DEGs.

### 2.4. Weighted Gene Coexpression Network Construction

The consensus DEGs were subjected to WGCNA [14, 22, 23]. The scale-free gene coexpression networks were constructed using the clinical features and prognostic information of TCGA-LUAD dataset and the WGCNA software package [15].

The appropriate soft threshold power was automatically estimated and generated for the standard scale-free network. The weighted adjacency matrix was constructed using the power function ADJ_*mn*_ = |COR_*mn*_|^*β*^ (COR_*mn*_ = Pearson's correlation between gene *m* and gene *n*, where ADJ_*mn*_ = adjacency between gene *m* and gene *n* and *β* is the soft thresholding parameter, which was used to transform adjacencies and correlations into a topological overlap matrix (TOM). The corresponding dissimilarity was calculated as 1-TOM. Module identification was carried out with the dynamic tree cut method by hierarchically clustering the genes using 1-TOM as the distance measure with a deep split value of 2 and a minimum size cutoff 50 for the resulting dendrogram. Highly similar modules were marked by clustering and merged with a height cutoff 0.25.

### 2.5. Identification of Clinical Feature Modules and Efficacy Evaluation of Pathological Stage Hub Genes

Module eigengenes (MEs), which are the first principal components in the PCA for each gene module, summarized the expression patterns of all genes into a single characteristic expression profile within a given module. The dynamic decision-making tree, node splitting method, and cluster analysis of the squared Euclidean distance were used to identify MEs related to these clinical features, especially those involved in the progression and prognosis of NSCLC. Modules with similar expression profiles were identified using the dynamic tree cut method. Highly similar modules were merged. Spearman's correlation analysis was carried out to confirm the object module, which was the most relevant module between the MEs and clinical traits. Depending on these, the module that had the highest absolute Spearman's correlation coefficient (PCC) value for the pathological stage and MEs was defined as the pathological stage module.

### 2.6. Identification, Characterization, and Validation of an mRNA Prognostic Model for NSCLC Patients

Association of genes in the pathological stage modules with survival of NSCLC patients was analyzed using a univariate Cox regression analysis. The genes with *P* value <0.05 were selected. A stepwise model selection by the Akaike information criterion (AIC) was further performed to avoid overfitting to select a final list of genes. A multivariate Cox hazard model analysis was performed to generate an mRNA prognostic signature model, which calculated the prognostic score as follows: prognostic score = ∑(*C* × EXP_mRNA_), where EXP is the fragments per kilobase million (FPKM) value of the mRNA and *C* is the regression coefficient for the corresponding mRNA in multivariate Cox hazard model analysis. The median prognostic score of the training dataset was used to differentiate high-risk group and low-risk group. Higher scores predicted higher risk. The prognostic performance of the mRNA signature model was measured using receiver operating characteristic (ROC) curves by comparing the area under the respective ROC curves (AUC). The mRNA signature was examined for its association with patient survival. Finally, the mRNA signature model was validated with an independent data set GSE11969 of NSCLC adenocarcinoma. All reported *P* values were two-sided. All analyses were carried out via the R/BioConductor (version 3.5.1). Survival curves and ROCs were generated by ggplot2, survival, and survivalROC packages.

## 3. Results

### 3.1. Identification of Consensus NSCLC DEGs in the Training Set and the Test Set

A total of 7 GEO datasets (GSE10072, GSE19188, GSE21933, GSE30219, GSE32863, GSE40275, and GSE7670) were selected from the 13 raw datasets after MetaQC quality control for subsequent analysis (Table 2 and Figure 2(a)). These datasets contained 590 NSCLC and 280 ANTs and were designated as the training set. In the training set, a total of 7373 DEGs were identified after filtering through the mean and standard deviation (SD) thresholds. A list of 7076 DEGs were subsequently obtained, and we eliminated batch effect after Fisher's *t* test and 300 permutations (Figure 2(b)). Hierarchical clustering of the seven datasets in the training set using the 7076 DEGs distinguished NSCLC from ANT samples (Figure 3(a)). In the TCGA-LUAD dataset which contained 20501 mRNAs in 517 NSCLC samples and 59 ANT samples, a total of 3592 DEGs were identified and designated as the test set. The DEGs in the test set distinguished NSCLC from ANT samples in the 2-way hierarchical cluster (Figure 3(b)). A total of overlapped 2146 DEGs between the training set and the test set were identified and designated as the consensus DEGs (Figure 3(c)).

### 3.2. Coexpression Network Construction and Identification of Modules Associated with Clinicopathological Features

We constructed a weighted gene coexpression network (WGCN) using the 2146 consensus DEGs and clinical traits and prognostic information from 515 NSCLC patients in the TCGA-LUAD test set. The results showed that the connections between the genes in the WGCN were in line with a scale-free network distribution (Figures 4(a)–4(d)). Modules with similar expression profiles were identified using the dynamic tree cut method (Figures 5(a) and 5(b)). Highly similar modules were merged (Figure 5(b)). A total of 14 WGCN modules ranging from 54 to 607 genes in each module were generated (Figure 5(c)). We further analyzed association of modules with clinicopathological features to identify pathological stage modules using Spearman's correlation and Module eigengenes analysis. The results showed the lightcyan module was most significantly associated with pathological M stage (*R* = 0.12, *P*=0.009), and this module contained 61 genes (Figure 5(c)).

### 3.3. Construction of an mRNA-Signature Prognostic Model and Characterization of Its Prognostic Performance Using NSCLC-LUAD

To investigate potential genes significantly associated with the survival of NSCLC patients, we performed a univariate Cox regression analysis using the lightcyan module genes. The results showed that the twelve genes *RRM2*, *RPS6KL1*, *RTL1*, *RXFP1*, *RRM1*, *RTCD1*, *RRAGB*, *RSPH10B2*, *RRM2B*, *RSPH9*, *RXFP2*, and *RUNX1* were significantly correlated with the overall survival of NSCLC patients (Table 3). We further performed a stepwise model selection by the Akaike information criterion (AIC), and six genes RRAGB, RSPH9, RPS6KL1, RXFP1, RTL1, and RRM2 were selected. Multivariate Cox hazard model analysis of association of these six genes with survival showed that RPS6KL1 and RXFP1 were independent factors associated with good overall survival in NSCLC patients, while RTL1 and RRM2 were independent factors associated with poor overall survival in NSCLC patients (Table 4). We generated an mRNA signature model which calculated the prognostic score: prognostic score = (−0.2491 × EXP_RRAGB_) + (−0.0679 × EXP_RSPH9_) + (−0.2317 × EXP_RPS6KL1_) + (−0.1035 × EXP_RXFP1_) + 0.1571 × EXP_RRM2_ + 0.1104 × EXP_RTL1_, where EXP is the FPKM value of the mRNA included in the model.

We characterized the prognostic performance of the six-mRNA signature model using the TCGA-LUAD dataset. According to prognostic scores, the median score was 0.972 and we separated NSCLC patients into the low-risk group (*n* = 253) and the high-risk group (*n* = 253) (Figure 6(a)). The high-risk group had significantly shorter survival time or lower survival probabilities than the low-risk group did (HR, 2.298; 95% CI, 1.711–3.086; log-rank test *P*=9.181 × 10^−9^) (Figure 6(b)). The area under ROC curve (AUC) was 0.994 or 0.776 in predicting the 1- to 10-year survival of NSCLC patients (Figure 6(c)). High expression of RRAGB, RSPH9, RPS6KL1, and RXFP1 and low expression of RTL1 and RRM2 predicted good survival (Figures 6(d)–6(i)). The results suggested that the six-mRNA signature could predict the prognosis of NSCLC-LUAD.

### 3.4. Validation of the Prognostic Performance of the Six-mRNA Signature in NSCLC Adenocarcinoma

To validate the prognostic performance of the six-mRNA model for NSCLC, we measured the prognostic performance of this model using the validation dataset GSE11969 of NSCLC adenocarcinoma. The results showed that the patients were divided into the high-risk group (*n* = 47) and the low-risk group (*n* = 47) according to the risk scores and the median cutoff point (Figure 7(a)). The high-risk group had significantly shorter survival time or lower survival probabilities than the low-risk group did (HR, 3.286; 95% CI, 1.79–6.03; log-rank test *P*=0.00013) (Figure 7(b)). The area under ROC curve in predicting 1- to 10-year survival of NSCLC was between 0.822 and 0.755 (Figure 7(c)). High expression of RRAGB, RSPH9, RPS6KL1, and RXFP1 and low expression of RTL1 and RRM2 expression predicted good survival of NSCLC patients (Figures 7(d)–7(i)). These results were consistent with those of the test set (compare Figures 6 and 7), supporting that the six-mRNA signature could predict the prognosis of NSCLC adenocarcinoma.

### 3.5. Relative Expression Levels of RRAGB, RSPH9, RPS6KL1, RXFP1, RRM2, and RTL1 in NSCLC Tissues and the High- and Low-Risk Groups

Examination of the expression patterns of these signature mRNAs revealed that RRAGB, RSPH9, and RXFP1 mRNA levels were significantly lower and RPS6KL1, RTL1, and RRM2 mRNA levels were significantly decreased in NSCLC of TCGA-LUAD, compared with the normal control (Figure 8(a)). The expression levels of RRAGB, RSPH9, RPS6KL1, and RXFP1 were significantly lower and RTL1 and RRM2 mRNA levels were significantly higher in the high-risk group than those in the low-risk group in NSCLC of TCGA-LUAD (Figure 8(b)). The expression levels of RRAGB, RSPH9, RPS6KL1, RXFP1, and RTL1 mRNA were significantly lower and the RRM2 mRNA level was significantly higher in the high-risk group than those in the low-risk group in NSCLC adenocarcinoma of GSE11969 (Figure 8(c)).

## 4. Discussion

In the current study, we have identified a six-gene prognostic model for NSCLC adenocarcinoma by calculating prognostic score using the formula: prognostic score = (−0.2491 × EXP_RRAGB_) + (−0.0679 × EXP_RSPH9_) + (−0.2317 × EXP_RPS6KL1_) + (−0.1035 × EXP_RXFP1_) + 0.1571 × EXP_RRM2_ + 0.1104 × EXP_RTL1_, where EXP is the FPKM value of the mRNA included in the model. Characterization of prognostic performance revealed that the model separates NSCLC patients in the TCGA-LUAD dataset into the low-risk score group and the high-risk score group with median prognostic score 0.972. Higher scores predicted higher risk. The area under ROC curve (AUC) was 0.994 or 0.776 in predicting the 1- to 10-year survival of NSCLC patients. The expression of each gene in the signature differentiates survival of NSCLC patients. The results were similar in the independent GSE11969 dataset of NSCLC adenocarcinoma. All these results support that the six-gene signature is an independent biomarker for prediction of overall survival of NSCLC adenocarcinoma.

Several expression-based gene signatures for NSCLC prognosis in the previous studies have been identified. The 8-gene signature (STAT1, CLU, GTSE1, NUSAP1, ABCA8, TNNT1, ENTPD3, and CPA3) can significantly stratify patients into low- and high-risk groups and predict patients in stage II-III benefiting from adjuvant chemotherapy [24]. The independent prognostic six-protein signature (c-SRC, Cyclin E1, TTF1, p65, CHK1, and JNK1) is identified for ADC and five-protein signature (EGFR, p38*α*, AKT1, SOX2, and E-cadherin) for SCC [25]. The 15-gene signature (ATP1B1, TRIM14, FAM64A, FOSL2, HEXIM1, MB, L1CAM, UMPS, EDN3, STMN2, MYT1L, IKBKAP, MLANA, MDM2, and ZNF236) can differentiate high- and low-risk subgroups with significantly different overall survival and is prognostic for both adenocarcinoma and squamous cell carcinoma cases [8]. The multigene RNA expression signature GeneFx® Lung classifies early-stage NSCLC patients as high-risk or low-risk for disease recurrence and predicts the overall survival [9]. The 50-gene signature novel scoring system is identified for tumor-infiltrating immune cells with strong correlation with clinical outcome of stage I/II non-small-cell lung cancer [26]. The 6-gene signature (*ABCC4*, *ADRBK2*, *KLHL23*, *PDS5A*, *UHRF1*, and *ZNF551*) is identified for independent prognosis of overall survival [10]. The Yin Yang Expression Ratio Signature containing 10 functionally opposing genes (*GRM1*, *IGFBP5*, *NRAS*, and *RECQL4* in the Yin group and *CRIP2*, *CD83*, *GATA2*, *HOXA5*, *SOSTDC1*, and *TNNC1* in the Yang group) significantly separates high- and low-risk patients with stage IA or IB adenocarcinoma and squamous cell carcinomas of all stages and can predict the benefit of adjuvant chemotherapy in high-risk patients with stage I NSCLC [11]. The 14-gene signature (11 cancer-related genes *BAG1*, *BRCA1*, *CDC6*, *CDK2AP1*, *ERBB3*, *FUT3*, *IL11*, *LCK*, *RND3*, *SH3BGR*, and *WNT3A* and three reference genes *ESD*, *TBP*, and *YAP1*) predicts survival in resected nonsquamous, non-small-cell lung cancer [4], identifies patients at high risk of mortality despite small, node-negative lung tumors [5], improves identification of patients at risk for recurrence in early-stage none small cell lung cancer [6], and predicts benefit from adjuvant chemotherapy for very early stage NSCLC and is superior over current NCCN criteria at identifying high-risk patients [7]. The 17-gene panel consisting of genes involved in epithelial-mesenchymal transition (EMT), hypoxia response, glycometabolism, and epigenetic modifications for non-small-cell lung cancer prognosis is identified through integrative epigenomic-transcriptomic analyses and clearly stratifies NSCLC patients with significant differences in overall survival [12]. Our six-gene prognostic signature for NSCLC adenocarcinoma include RRAGB, RSPH9, RPS6KL1, RXFP1, RRM2, and RTL1 genes which are not contained in the previous gene signatures. Therefore, our six-gene signature is likely a novel tool for NSCLC adenocarcinoma prognosis.

Our data indicated that high expression of RRAGB, RSPH9, RPS6KL1, and RXFP1 and low expression of RTL1 and RRM2 predicted good survival. Among these six genes, we found that RRM2 (ribonucleotide reductase regulatory subunit M2 and ribonucleoside-diphosphate reductase subunit M2) is overexpressed in NSCLC tissues. The RRM2 mRNA levels are higher in the high-risk group than those in the low-risk group and may differentiate the survival of NSCLC patients. Studies have shown that RRM2 is known as a marker that may be involved in predicting clinical response to gemcitabine plus docetaxel [27] and predicting the treatment response to platinum-based chemotherapy and survival [28, 29] in non-small-cell lung cancer patients. The expression levels of RRM2 and differences between primary tumors and infiltrated regional lymph nodes were correlated with relapse-free survival (RFS) and overall survival (OS) in patients with resectable non-small-cell lung cancer [30]. RRM2 regulates antiapoptotic protein Bcl-2 in head and neck and lung cancers [31, 32]. BRCA1-regulated RRM2 expression protects glioblastoma cells from endogenous replication stress and promotes tumorigenicity [33]. RRM2 is regulated by the transforming growth factor beta regulator 4 (TBRG4) gene which affects tumorigenesis in human H1299 lung cancer cells [34]. It is likely that RRM2 plays an essential role in NSCLC development and progression and may serve as a key marker for NSCLC prognosis.

The model signature genes RSPH9, RPS6KL1, RXFP1, and RTL1 have been revealed to be involved in cancer activity. RSPH9 (radial spoke head 9 homolog) was significantly hypermethylated and downregulated in the hepatocellular carcinoma (HCC) and epigenetic silencing of RSPH9 may be associated with hepatocellular carcinoma [35]. In multivariate regression analysis, hypermethylation of RSPH9 was an independent predictor of non-muscle invasive bladder cancer (NMIBC) recurrence and progression, and RSPH9 could be of value for the assessment of disease recurrence and progression and for clinical decision-making regarding treatment [36]. RPS6KL1 (ribosomal protein S6 kinase-like 1) mutation hot spots were confirmed and validated in colorectal cancers with microsatellite instability, which might be used to develop personalized tumor profiling and therapy [37]. RXFP1 (relaxin family peptide receptor 1, relaxin receptor 1, and relaxin/insulin-like family peptide receptor 1) is a G protein-coupled receptor with the extracellular low-density lipoprotein A (LDL-A) module located at the N-terminus. Studies have revealed that RXFP1 is activated by both C1q-tumor necrosis factor-related protein 8 (CTRP8) and relaxin and contributes to growth and invasion of human glioblastoma [38–40]. Suppression of RXFP1 inhibits prostate cancer tumorigenesis, growth, and metastasis [41–43]. Relaxin 2/RXFP1 Signalling induces cell invasion via the beta-catenin pathway in endometrial cancer [44]. Expression of RXFP1 is decreased in idiopathic pulmonary fibrosis [45] and mediates the effects of miR-144-3p in lung fibroblasts from patients with idiopathic pulmonary fibrosis [46]. RXFP1 protects against airway fibrosis during homeostasis but not against fibrosis associated with chronic allergic airways disease [47]. RTL1 (retrotransposon-like protein 1, retrotransposon Gag like 1, also known as Peg11, paternally expressed 11) is essential for maintenance of the fetal capillaries. Both its loss and its overproduction cause late-fetal and/or neonatal lethality in mice [48]. The Rtl1 promoter is hypermethylated in the placentas with fetal growth restriction. Infants with severe SGA have abnormal placental DNA methylation of CpG1 in the CG4 region of RTL1, suggesting the existence of disturbed epigenetic control in utero [49]. Overexpression of RTL1 in melanoma cells accelerated cutaneous melanoma cell proliferation, promoted the passage of the cell cycle beyond G1 phase, and increased the expression of cell cycle related genes, and RTL1 promotes melanoma cell proliferation by regulating the Wnt/*β*-Catenin signalling pathway [50]. RTL1 activation serves as a driver of HCC. Overexpression of RTL1 was detected in 30% of analyzed human HCC samples, indicating the potential relevance of this locus as a therapeutic target for patients [51]. RRAGB (Ras related GTP binding B) mediates mTOR (mechanistic target of rapamycin kinase) and TRIM37 (tripartite motif containing 37) pathways related to amino acid-stimulated MTORC1 (MTOR complex 1) signalling and autophagy [52]. In the current study, we found that RRAGB, RSPH9, RPS6KL1, RXFP1, and RTL1 are differentially expressed between NSCLC and ANTs. Expression of RRAGB, RSPH9, RPS6KL1, RXFP1, and RTL1 is significantly associated with survival of NSCLC. These results suggest that RRAGB, RSPH9, RPS6KL1, RXFP1, and RTL1 may be key factors in NSCLC activity.

## 5. Limitations

(1) The relative expression profiles of RTL1 expression in the TCGA-LUAD and GSE11969 of NSCLC adenocarcinoma are not consistent. This may be due to intervariation between different detection platforms. (2) The six-gene prognostic signature remains to be evaluated for clinical application using multicenter randomized controlled studies and mechanistic investigation using in vivo and in vitro experiments.

## 6. Conclusions

In summary, we have identified a six-gene prognostic model for NSCLC adenocarcinoma by calculating prognostic-score using the formula: prognostic score = (−0.2491 × EXP_RRAGB_)+ (−0.0679 × EXP_RSPH9_) + (−0.2317 × EXP_RPS6KL1_) + (−0.1035 × EXP_RXFP1_) + 0.1571 × EXP_RRM2_ + 0.1104 × EXP_RTL1_, where EXP is the FPKM value of the mRNA included in the model. This signature and the genes RRAGB, RSPH9, RPS6KL1, RXFP1, RRM2, and RTL1 included in this model are independent biomarkers for prediction of overall survival of NSCLC adenocarcinoma. The role of the signature genes played in NSCLC adenocarcinoma activity and prognosis remains to be investigated in the future.

## Figures and Tables

**Figure 1:** Workflow of the integrated analysis and WGCNA analysis of the NSCLC datasets. Figure 1 was reproduced from Sun et al. [16].

**Figure 2:** Meta-analysis of differentially expressed genes involved in NSCLC by combining *P* values. (a) Principal component analysis (PCA) biplot of quality control measures in thirteen NSCLC studies. (b) The number of differentially expressed genes plotted as a function of false discovery rate (FDR) in the analysis of four different datasets and four different meta-analysis algorithms (maxP, minP, roP, and adaptively weighted statistic). Figure 2 was reproduced from Sun et al. [16].

**Figure 3:** Identification of consensus DEGs in the training and the test datasets of NSCLC patients. (a) Heat map and two-way hierarchical clustering based on 7076 DEGs that were differentially expressed between NSCLC and ANT samples of the training set. ANT (green label) and NSCLC (red label) samples fell into separate clusters. (b) The 3592 DEGs NSCLC (red label) vs. ANT (blue label) of the TCGA-LUAD test set. Each column represents a sample, and each row represents the mRNA level. The color scale represents the raw *Z*-score ranging from blue (low expression) to red (high expression). Dendrograms beside each heat map correspond to the hierarchical clustering of the 3592 DEGs by the expression level. (c) A Venn diagram showing the overlap of DEGs detected in the training and test sets. Figure 3 was reproduced from Sun et al. [16].

**Figure 4:** Determination of parameter *β* of the adjacency function in the weighted gene correlation network analysis (WGCNA) algorithm. (a) Analysis of the scale-free fit index for various soft thresholding powers *β*. (b) Analysis of the mean connectivity for various soft thresholding powers. (c) Histogram of connectivity distribution when *β* = 19. (d) Checking the scale-free topology when *β* = 19. Figure 4 was reproduced from Sun et al. [16].

**Figure 5:** Network construction of the weighted coexpressed genes and their associations with clinical traits. (a) Hierarchical clustering tree of the TCGA-LUAD samples based on the DEGs. Dendrogram tips are labeled with the TCGA-LUAD unique name and experiment identifier. In the hierarchical dendrogram, lower branches correspond to higher coexpression (height = Euclidean distance). Identical colors in the ten bands below the dendrogram depict the TCGA-LUAD clinical traits. (b) Heat map view of topological overlap of coexpressed genes in different modules. The heat map was generated from the topological overlap values between genes. The genes were grouped into modules labeled by a color code, which are given under the gene dendrogram on both sides. The topological overlap was high among genes of same module. (c) Module-trait relationships for gender, histological type, lymphatic invasion, tumor status, treatment condition, and pathologic stage. Numbers shown represent Pearson correlations between the modules and traits. *P* values are in parentheses. Numbers on the color bar refer to the strength of the correlation in the table (red = 1, blue = −1). *T*, extent of the tumor; *N*, extent of spread to the lymph nodes; *M*, presence of metastasis. Figure 5 was reproduced from Sun et al. [16].

**Figure 6:** The prognostic performance of the six-gene signature in the TCGA-LUAD test cohort. (a) Risk score analysis of the six-gene signature of NSCLC. Risk score of gene signature (top); duration of cases (middle); low and high score groups for the six genes (bottom). (b) Survival analysis of the high-risk group and the low-risk group using Kaplan–Meier curves. (c) The prognostic efficiency of the six-gene signature for survival time. ROC curves of the six-gene signature for predicting 1- to 10-year survival were analyzed. (d–i) The independent prognostic efficiency of individual mRNA in the six-gene signature of the test set. (d) RRM2; (e) RPS6KL1; (f) RTL1; (g) RXFP1; (h) RRAGB; (i) RSPH9. Horizontal axis, overall survival time. Vertical axis, overall survival.

**Figure 7:** The prognostic performance of the six-gene signature in the GSE11969 validation cohort. (a) Risk score analysis of the six-gene signature of NSCLC. Risk score of gene signature (top); duration of cases (middle); low and high score groups for the six genes (bottom). (b) Survival analysis of the high-risk group and the low-risk group using Kaplan–Meier curves. (c) The prognostic efficiency of the six-gene signature for survival time. ROC curves of the six-gene signature for predicting 1- to 10-year survival were analyzed. (d–i) The independent prognostic efficiency of individual mRNA in the six-gene signature in the validation set. (d) RRM2; (e) RPS6KL1; (f) RTL1; (g) RXFP1; (h) RRAGB; (i) RSPH9. Horizontal axis, overall survival time. Vertical axis, overall survival.

**Figure 8:** The relative levels of RRAGB, RSPH9, RPS6KL1, RXFP1, RRM2, and RTL1 in NSCLC adenocarcinoma. (a) Compared with the normal control, RRAGB, RSPH9, and RXFP1 mRNA levels were significantly decreased and RPS6KL1, RTL1, and RRM2 mRNA levels were significantly increased in NSCLC of TCGA-LUAD. (b) The expression levels of RRAGB, RSPH9, RPS6KL1, and RXFP1 were significantly lower and RTL1 and RRM2 mRNA levels were significantly higher in the high-risk group than those in the low-risk group of TCGA-LUAD. (c) The expression levels of RRAGB, RSPH9, RPS6KL1, RXFP1, and RTL1 were significantly lower and RRM2 mRNA levels was significantly higher in the high-risk group than those in the low-risk group in NSCLC adenocarcinoma of GSE11969.

**Table 1:** Characteristics of the public microarray datasets used in this study.

Study	Species/array platform	Samples	Number of samples	Set
GSE19188	[HG-U133_Plus_2] Affymetrix Human Genome U133 Plus 2.0 Array(GPL570)	NSCLC vs. control tissue	NSCLC = 91 (LUAD 45, LUSC 46), control tissue = 65, total = 156	Training set
GSE30219	[HG-U133_Plus_2] Affymetrix Human Genome U133 Plus 2.0 Array(GPL570)	NSCLC vs. control tissue	NSCLC = 293, control tissue = 14, total = 307	Training set
GSE10072	[HG-U133A] Affymetrix Human Genome U133A Array (GPL96)	NSCLC vs. control tissue	NSCLC = 58 (LUAD 58), control tissue = 49, total = 107	Training set
GSE7670	[HG-U133A] Affymetrix Human Genome U133A Array (GPL96)	NSCLC vs. control tissue	NSCLC = 28 (LUAD 28), control tissue = 30, total = 58	Training set
GSE2514	[MG_U74Av2] Affymetrix Murine Genome U74A Version 2 Array (GPL81)	NSCLC vs. control tissue	NSCLC = 20, control tissue = 19, total = 39	Training set
GSE32863	Illumina HumanWG-6 v3.0 expression beadchip (GPL6884)	NSCLC vs. control tissue	NSCLC = 58 (LUAD 58), control tissue = 58, total = 116	Training set
GSE21933	Phalanx Human OneArray (GPL6254)	NSCLC vs. control tissue	NSCLC = 21, control tissue = 21, total = 42	Training set
GSE40275	Human Exon 1.0 ST Array (GPL15974)	NSCLC vs. control tissue	NSCLC = 41, control tissue = 43, total = 84	Training set
GSE12472	Agilent-012391 Whole Human Genome Oligo Microarray G4112A (Feature Number version) (GPL1708)	NSCLC vs. control tissue	NSCLC = 35 (LUSC 35), control tissue = 28, total = 63	Training set
GSE80796	[HuGene-1_0-st] Affymetrix Human Gene 1.0 ST Array [transcript (gene) version] (GPL6244)	NSCLC vs. control tissue	NSCLC = 309, control tissue = 196, total = 505	Training set
GSE8500	Human 3.0 A1 (GPL3991)	NSCLC vs. control tissue	NSCLC = 40, control tissue = 8, total = 48	Training set
GSE85841	Agilent-067406 Human CBC lncRNA + mRNA microarray V4.0 (GPL20115)	NSCLC vs. control tissue	NSCLC = 8, control tissue = 8, total = 16	Training set
GSE19027	[HG-U133A] Affymetrix Human Genome U133A Array (GPL96)	NSCLC vs. control tissue	NSCLC = 21, control tissue = 39, total = 60	Training set
TCGA-LUAD	Human Illumina HiSeq 2000	LUAD vs. control tissue	LUAD = 517, control tissue = 59, total = 576	Test set
GSE11969	Agilent Homo sapiens 21.6 K custom array (GPL7015)	Overall survival	LUAD = 94, Overall survival information = 94	Validation set

GSE, Gene Expression Omnibus accession number; TCGA, the Cancer Genome Atlas; NSCLC, non-small-cell lung cancer; LUAD, lung adenocarcinomal; LUSC, lung squamous cell carcinoma.

**Table 2:** Quality control of the training datasets.

No.	Datasets	IQC	EQC	CQCg	CQCp	AQCg	AQCp	Rank
1	GSE19188	8.56	2^*∗*^	307.65	160.1	0.79^*∗*^	54.72	2.33
2	GSE30219	4.43	2^*∗*^	307.65	182.57	0.76^*∗*^	71.49	2.58
3	GSE10072	9.76	2^*∗*^	307.65	178.14	0.14^*∗*^	49.61	3.67
4	GSE7670	6.48	1.7^*∗*^	307.65	133.26	0.2^*∗*^	43.06	4.75
5	GSE2514	3.66	1.53^*∗*^	307.65	111.14	0.4^*∗*^	22.46	5.67
6	GSE32863	5.73	1.7^*∗*^	307.65	63.92	0.08^*∗*^	32.71	5.75
7	GSE21933	4.43	1^*∗*^	307.65	52.67	0.37^*∗*^	23.99	6.08
8	GSE40275	3.96	1.53^*∗*^	8.68	34.36	0.29^*∗*^	21.19	7.50
9	GSE12472	0.24^*∗*^	1.53^*∗*^	7.06	44.83	0.32^*∗*^	12.49	8.33
10	GSE80796	2.08^*∗*^	1.05^*∗*^	0.27^*∗*^	2.32^*∗*^	0.28^*∗*^	1.38^*∗*^	10.00
11	GSE8500	3.51	0.4^*∗*^	0.38^*∗*^	4.02	0.26^*∗*^	0.06^*∗*^	10.67
12	GSE85841	0.04^*∗*^	0.62^*∗*^	0.71^*∗*^	0.31^*∗*^	0.04^*∗*^	0.26^*∗*^	11.67
13	GSE19027	1.35^*∗*^	0.39^*∗*^	0^*∗*^	7.83	0.03^*∗*^	0.24^*∗*^	12.00

NSCLC, non-smal-cell lung carcinoma; GSE, GEO dataset; IQC, internal quality control indexes; EQC, external quality control indexes; CQCg and CQCp, consistency of differential expression quality control indexes for genes and pathways; AQCg and AQCp, accuracy quality control indexes for genes and pathways. ^*∗*^*P* value not significant after Bonferroni correction.

**Table 3:** Univariate Cox regression analysis of lightcyan module genes and overall survival^*∗*^.

Genes	Overall survival		
	HR	CI (95% CI)	*P* value
RRM2	1.291	1.152–1.448	<0.001
RPS6KL1	0.798	0.709–0.897	<0.001
RTL1	1.132	1.054–1.215	0.001
RXFP1	0.864	0.787–0.949	0.002
RRM1	1.438	1.121–1.845	0.004
RTCD1	1.489	1.100–2.014	0.010
RRAGB	0.706	0.537–0.929	0.013
RSPH10B2	0.909	0.842–0.981	0.014
RRM2B	0.784	0.641–0.958	0.017
RSPH9	0.901	0.826–0.983	0.019
RXFP2	0.734	0.562–0.960	0.024
RUNX1	0.798	0.645–0.988	0.038

HR, hazard ratio; CI, confidence interval. ^*∗*^Association of the 61 genes of the lightcyan module with survival was analyzed using univariate Cox regression analysis. Presented in the table were those which showed significant association (*P* < 0.05).

**Table 4:** Multivariate Cox regression analysis of lightcyan module genes and overall survival^*∗*^.

Genes	*β*	HR	selogHR	*z*	CI (95% Cl)	*P*
RRAGB	−0.2491	0.7795	0.1360	−1.83	0.5971–1.0176	0.06700
RSPH9	−0.0679	0.9344	0.0462	−1.47	0.8535–1.0230	0.14201
RPS6KL1	−0.2317	0.7932	0.0608	−3.81	0.7042–0.8935	0.00014^#^
RTL1	0.1104	1.1167	0.0380	2.91	1.0367–1.2030	0.00364^#^
RXFP1	−0.1035	0.9016	0.0497	−2.08	0.8180–0.9939	0.03720^#^
RRM2	0.1571	1.1701	0.0626	2.51	1.0350–1.3229	0.01209^#^

^*∗*^The listed genes were selected by the Akaike information criterion (AIC) model from the significant genes after the univariate Cox regression analysis (Table 3). Multivariate Cox regression analysis of association of the listed genes with survival was performed to reveal the independent predictor for survival and generate a prognostic risk score model. *β*, regression coefficient; HR, hazard ratio; CI, confidence interval; ^#^*P* < 0.05.

## Data Availability

The data used to support the findings of this study are included within the article.

## Abbreviations

LC: Lung cancer
NSCLC: Non-small-cell lung cancer
ANT: Adjacent normal tissue
WGCNA: Weighted gene coexpression network analysis
TCGA: The Cancer Genome Atlas
DEGs: Differentially expressed genes
HR: Hazard ratio
AUC: Area under the curve
GEO: Gene Expression Omnibus
GSE: Gene expression data series
LIMMA: Linear models for microarray analysis
QC: Quality control
SD: Standard deviation
TOM: Topological Overlap Matrix
ME: Module eigengene
KEGG: Kyoto Encyclopedia of Genes and Genomes
AJCC: American Joint Committee on Cancer
PCC: Pearson's correlation coefficient
PCA: Principal component analysis
ROC: Receiver operating characteristic
David: The Database for Annotation, Visualization, and Integrated Discovery
LUAD: Lung adenocarcinoma
NCCN: National Comprehensive Cancer Network
EMT: Epithelial-mesenchymal transition
FPKM: Fragments per kilobase million.
